# Assessment of Antioxidative and Alpha-Amylase Potential of Polyherbal Extract

**DOI:** 10.1155/2022/7153526

**Published:** 2022-05-31

**Authors:** Mohsina Patwekar, Faheem Patwekar, Amine Mezni, Syed Sanaullah, Shaikh Rohin Fatema, Ustad Almas, Irfan Ahmad, Vineet Tirth, Jewel Mallick

**Affiliations:** ^1^Luqman College of Pharmacy, Gulbarga, Karnataka, India; ^2^Department of Chemistry, College of Science, Taif University, P.O. Box 11099, Taif 21944, Saudi Arabia; ^3^Department of Clinical Laboratory Sciences, College of Applied Medical Sciences, King Khalid University, Abha, Saudi Arabia; ^4^Mechanical Engineering Department, College of Engineering, King Khalid University, Abha 61421, Asir, Saudi Arabia; ^5^Department of Pharmacy, BGC Trust University Bangladesh, Chittagong 4381, Bangladesh

## Abstract

The present study aims to prepare a polyherbal formulation (PHF) of *Azadirachta indica* (Neem), *Aloe barbadensis* (Aloe vera), *Allium sativum* (garlic), *Acacia arabica* (Babul), and *Aegle marmelos* (Bel) and evaluation of antidiabetic and antioxidant activity utilizing the in vitro model. Air-dried powder of 5 medicinal plants, which are divided into equal portions, and PHF, is prepared by the soxhlet technique using polar and nonpolar solvents. The PHF is screened for the phytochemical screening, and then the antidiabetic activity is determined by alpha-amylase inhibition. The extracts thus obtained are also subjected to the inhibition assay by the use of (DNS) dinitro salicylic acid. The antioxidant activity was determined by the DPPH radical scavenging assay, H_2_O_2_ scavenging assay, and TBARS assay. In in vitro study, the result revealed polyherbal formulation in which hot water extract has the topmost inhibitory effect on alpha-amylase activity, ranging from 20.4% to 79.5% with an IC50 value of 48.98 ± 0.31 *μ*g/ml. This extract clearly showed the effective lowering of postprandial hypertriglyceridemia (PPHG). In the antioxidant activity carried out by using the (DPPH) radical scavenging assay, the highest result was obtained by the concentration of 250 *μ*g/ml, which was around 77.2 ± 0.05 with statistical significance compared with control (a: *p* < 0.01; b: *p* < 0.001), while in the GTA method, the highest result was obtained by the concentration of 250 *μ*g/ml, which was around 78.2 ± 0.05, and in the case of the TBARS assay, the concentration of 250 *μ*g/ml gave around 76.2 ± 0.03 anti-oxidant value. In conclusion, the study shows that polyherbal formulation has superior antidiabetic activity and antioxidant properties.

## 1. Introduction

DM is a systemic metabolic disorder characterized by hyperglycemia, hyperlipidemia, hyperaminoacidemia, and hypoinsulinemia in which insulin action and insulin production both are reduced [1]. Treatment of diabetes depends on its etiology and is primarily divided into two types. Type I (IDDM) is insulin-dependent diabetes mellitus and is commonly known as “juvenile-onset.” In type I, the body does not produce any type of insulin production. Approximately 5–10% of human beings suffer from this type of DM. Type II (NIDDM) is a noninsulin-dependent diabetes mellitus in which the body tissues do not respond to insulin, resulting in hyperglycemia. In 2011, the International Diabetes Federation (IDF) estimated the total prevalence of DM at 366 million, and it assumes that, in 2030, it will increase to 550 million [2–4]. There are top 5 reasons for death worldwide, one of them is DM, and about 6 people die from complications of diabetes every minute [5]. WHO estimates (2002) that 7.1 million people worldwide die from hypertension, 4.4 million from hypercholesterolemia, and 2.6 million from obesity. In adults, type II DM is more common than type I DM [6–8]. Natural antioxidants observed in plants involve tannins, flavonoids, vitamin C (ascorbic acid), and vitamin E (alpha-tocopherol). They may protect against diabetes-induced cellular damage and reactive oxygen species (ROS) production [9].

Botanical studies of conventional natural medicines show approximately around 1,200 species have been used for diagnosis as well as treatment of hyperglycemia [10]. Different combinations of polyherbal-based therapy are playing a critical role in the cure of type II DM and are correlated with other diseases [11]. The World Health Organization has indexed species of 21,000 flora, which might be utilized for remedial purposes around the world [12]. In India, there are 2500 species of which approximately 800 have been suggested to show antidiabetic activity [13]. *Azadirachta indica* leaf extract confirmed the reduction of peripheral utilization of glucose and glycogenolytic impact [14]. It also blocks the inhibitory effects of serotonin on glucose-mediated insulin secretion [15].

*Aloe vera* extract contains active compounds such as vitamins, minerals, enzymes, organic acids, polysaccharides, and phenolic compounds. It has been stated that the polysaccharides present in the *Aloe vera* extract have anti-inflammatory, antidiabetic, antioxidant, and antiaging properties [16, 17]. *Acacia arabica* is found throughout India, especially in the west. The herbal extract acts as an antidiabetic agent, and it is used as an agent that increases insulin secretion [18]. Oral administration of *Allium Sativa* extract significantly reduced serum glucose, total cholesterol, triglyceride, urea, uric acid, creatinine, AST, and ALT levels [19]. *Aegle marmelos* leaf extract is being utilized in Ayurveda as a medicinal drug for diabetes. A methanolic extract of *Aegle marmelos* extracts was discovered to drop glucose levels in alloxan diabetic rats. Oxidative stress produced by means of alloxan change is determined to be considerably reduced by the administration of *Aegle marmelos* extract (Figure 1) [20].

The idea of polyherbal formulation (PHF) is amazing in the therapeutic system. Traditional Indian medicine uses complex herbal preparations and herbal concentrations rather than individual herbal preparations. The traditional restorative in India is called Ayurveda, and Ayurvedic herbs come in a variety of formulations, most of which contain PHF. Because PHF is a natural product, it is relatively inexpensive, environmentally friendly, and more readily available than homoeopathic remedies. Increasing availability and affordability are driving demand worldwide, where expensive modern treatment is not. [21]. Polyherbal formulations combine several herbs carefully in selected portions to increase the therapeutic efficacy and reduce toxicity [22].

## 2. Materials and Methods

### 2.1. Instruments and Chemicals

Soxhlet apparatus was used for the extraction process of the different herbs. The solvents or chemicals used in this procedure are hexane, benzene, chloroform, hot water, and cold water. PPA (porcine pancreatic amylase) and acarbose were purchased and procured from a lab trading laboratory in Aurangabad, Maharashtra, India. All chemicals used were of analytical grade.

### 2.2. Plant Materials

Based on this background information, the main aim of this study is to assess the antidiabetic activity and alpha-amylase inhibition of polyherbal formulation Herbal composition of selected plants has been mentioned in Table 1.

### 2.3. Sample Collection

The plant sample was collected and authenticated by the botanist, Dr. Madhava Chetty, Department of Botany, Sri Venkateswara University, Tirupati, India.

### 2.4. Sample Preparation

The parts of the plant were washed with water and dried in the shade. Dried samples were powdered by using a grinder. The composition is prepared by adding all the ingredients in equal portions, mixing thoroughly until homogeneity is obtained and storing in a sealed container until extraction.

### 2.5. Preparation of Polyherbal Formulations (PHF)

The PHF extract was prepared by using a Soxhlet extractor. The herbal powder composition was successively extracted with polar and nonpolar solvents. The solvents used were hexane, benzene, chloroform, ethanol, hot water, and cold water.

#### 2.5.1. Cold Water Extract

Cold water extract was prepared by the addition of distilled water to the grounded product in a 1 : 5 ratio and put in a rotary shaker at 37°C, 120 rpm for a day. After a day, the filtered extract is stored in the refrigerator.

#### 2.5.2. Hot Water Extract

Hot water extract was prepared by adding 400 ml of hot distilled water to 100 gm of herbal powder.

#### 2.5.3. Successive Solvent Extraction

Similarly, bioactive compounds were extracted from drug powder with organic solvent in a ratio of 1 : 4 according to the Soxhlet method. The resulting crude extract was transferred to a vial and kept in a cold storage box for future study.

### 2.6. In Vitro PPA Inhibition Assay

DNS analysis: alpha-amylase inhibition was determined by measuring the reducing sugar released in this assessment. The inhibitory activity of the enzyme was shown as a reduction in the released unit of glucose [23]. Plant extracts with a concentration starting from 10–100 *μ*g have been incubated with 1 ml of 1-unit PPA enzyme for 30 minutes at 37°C. After incubation with 1 ml of 1% buffered starch, the combination is subjected to further incubation for 10 minutes at RT (room temperature). The reaction was stopped by adding 1 ml of DNS reagent, and the contents have been heated in a boiling water tube for 5 minutes. A blank is obtained with the absence of plant extract, and the enzyme is replaced with an equal amount of 0.1 M phosphate buffer. A control representing 100% enzyme activity without plant extract was also included. The absorbance was studied at 540 nm in a UV spectrometer. The reducing sugar released from starch was estimated as glucose equivalent from the standard graph. Acarbose is a standard antidiabetic drug used as a +ve control for studying the inhibition of alpha-amylase antidiabetic property. The % of inhibition can be expressed by the inhibition of alpha-amylase and calculated by a formula which is given as follows:

(1) $$\begin{array}{c} \%\text{ inhibition}=\frac{\text{absorbance of control}-\text{absorbance of test}}{\text{absorbance of }{\text{control}}^{*}}. \end{array}$$

The IC50 value of acarbose and PHF extract of various solvents has been studied from the graph of % of inhibition vs. concentration (*μ*g/ml). IC50 value is described as the concentration of extract needed to inhibit 50% of PPA activity.

### 2.7. Antioxidant Activity

Antioxidant activity of polyherbal formulation has been calculated by the DPPH radical scavenging assay [24], the GTA (green tea antioxidants) activity [25], and by using the thiobarbituric acid reactive substance assay (TBARS) [26].

### 2.8. Statistical Analysis

All assays were performed at least in triplicate, and the results were expressed as mean ± standard deviation (SD). Differences were evaluated by the one-way analysis of variance (ANOVA) test completed by Tukey's multicomparison test. Differences were considered significant at *p*.

## 3. Results

### 3.1. Preliminary Phytochemical Screening

Qualitative phytochemical screening revealed the presence of carbohydrates, glycosides, alkaloids, steroids, terpenoids, flavonoids, phenol, tannins, and saponins as shown in Table 2.

### 3.2. Alpha-Amylase Activity

In the present analysis of polyherbal formulation, PHF extract of five different chemicals enabled a greater drop, that is, a reduction in alpha-amylase activity. Acarbose is a standard antidiabetic drug that has +ve control at concentrations of 10–100 ug/ml as shown by procaine pancreatic alpha-amylase assay inhibitory activity from 15.65% to 55.30% with an IC50 value of 90.35 ± 0.20 ug/ml (Table 3, Figure 2). Polyherbal formulation 1 hot water extract shows topmost inhibitory effect on alpha-amylase activity from 20.4% to 79.5% with an IC50 value 48.98 ± 0.31 *μ*g/ml (Table 4, Figure 3), PHF ethanol, cold water extract, benzene, and hexane extract at the concentrations of 10–100 *μ*g/ml revealed a moderate inhibitory effect on alpha-amylase activity from 14.6% to 68.6%, 23.3% to 53.4%, 38.17% to 55.9%, and 9.6% to 36.6% respectively, with IC50 values 69.42 ± 0.25 ug/ml, 90.55 ± 0.35 ug/ml, and 72.86 ± 0.28 Ug/ml, respectively (Tables 5–8, Figures 4–7).

### 3.3. Antioxidant Activity

In DPPH radical scavenging assay, the PHF activates at different concentrations as shown in Figure 8(a) and Table 9. It is compared with standard ascorbic acid as a reference. It is revealed to be the most effective DPPH radical scavenging assay at concentration. The range starts from 50 *μ*g/ml to 250 *μ*g/ml. The highest result was obtained by the concentration of 250 *μ*g/ml, which was around 77.2 ± 0.05 with statistical significance compared with control (a: *p* < 0.01; b: *p* < 0.001).

In the GTA method, the PHF activity at different concentrations, as shown in Figure 8(b) and Table 10 compared with standard ascorbic acid, show H_2_O_2_ decomposition activity in a dose-dependent way, estimated at 250 *μ*g/ml. The highest result was obtained by the concentration of 250 *μ*g/ml, which was around 78.2 ± 0.05 with statistical significance compared with control (a: *p* < 0.01, b: *p* < 0.001).

In the TBARS assay, the % inhibition of PHF at different concentrations indicates that the PHF can probably inhibit lipid peroxidation in a dose-dependent manner when compared with herbal extracts. The highest result was obtained by the concentration of 250 *μ*g/ml, which was around 76.2 ± 0.03 with statistical significance compared with control (a: *p* < 0.01; b: *p* < 0.001) as shown in Figure 8(c) and Table 11.

## 4. Discussion

The PHF is assessed for their particular alpha-amylase inhibitory assay. The result shows that PHF (1) hot water extract has the best inhibitory impacts on alpha-amylase with an IC50 90.35 ± 0.20, which is comparatively less than acarbose, indicating that PHF hot extract has better activity because of the presence of phytochemicals that act as potential alpha-amylase inhibitors including glycosides, steroids, phenol, triterpenoids, and others. In the antioxidant activity carried out by using the DPPH radical scavenging assay, the highest result was obtained by the concentration of 250 *μ*g/ml, which was around 77.2 ± 0.05 with statistical significance compared with control (a: *p* < 0.01; b: *p* < 0.001), while in the results obtained in the GTA method, the highest result was obtained by the concentration of 250 *μ*g/ml which was around 78.2 ± 0.05, and in the case of the TBARS assay, the concentration of 250 *μ*g/ml gave around 76.2 ± 0.03 antioxidant value.

In comparison with the individual herb, the PHF has the best antioxidant remedy capability, especially for diabetic mellitus [27]. In the present investigation, the polyherbal formulation was prepared with *Azadirachta indica* (neem), A*loe barbadensis* (*Aloe vera*), *Allium sativum* (garlic), *Aegle marmelos* (bel), and *Acacia arabica* (babul). The study assessed the antioxidant activity of PHF and individual plant extracts through DPPH free radical scavenging and the TBARS test. DPPH is a constant, nitrogen-focused free radical [28]. Our research showed that the antioxidant ability of PHF changed to a greater extent compared to a single plant extract. Some results have shown direct correspondence between general phenolic content and antioxidant interest. The organic composition and chemical structure of active additives of the extract are good factors contributing to the acceptability of natural antioxidants [14]. The alpha-amylase inhibitors are utilized as adjuvant dietary supplements that determine the assimilation and ingestion of carbohydrates. Simultaneously, artificial inhibitor's purpose has numerous side consequences, including abdominal ache, diarrhea, and smooth faces in the colon [29]. Herbal combinations are used in India's conventional medicine method, and our PHF extract has good alpha-amylase activity [30].

## 5. Conclusion

In this conclusion, the polyherbal formulation is made with 5 medicinal plants that are *Azadirachta indica, Aloe barbadonsis, Allium sativum, Acacia arabica, and Aegle marmelos,* containing secondary metabolites and bioactive components that have therapeutic potential. The result obtained suggests that PHF of hot water extract is stated to have greater bioactive components. The interest of alpha-amylase enzyme therapy can be utilized as an oral hypoglycemic agent to control PPHG.

### 5.1. Future Prospects

A number of studies have shown that polyherbal formulations have strong antidiabetic efficacy in various animal models. To create a formulation's safety profile, toxicology tests on the described polyherbal formulations are required. At the molecular level, the mechanism of action of polyherbal formulations' antidiabetic efficacy should be investigated. It ensures that polyherbal compositions have a high level of pharmacological activity. In addition, pharmacokinetic and pharmacodynamic studies for the disclosed polyherbal formulation can be carried out. Clinical trials for polyherbal formulations with superior therapeutic and nontoxic effects can be conducted. As a result, patent applications for polyherbal compositions can be submitted to the patent office. A new and improved antidiabetic polyherbal formulation will be introduced to the market to replace the synthetic antidiabetic medication that has been linked to serious side effects.

## Figures and Tables

**Figure 1:** (a) *Azadirachta indica* (neem), (b) *Aloe barbadensis* (*Aloe vera*), (c) *Allium sativum* (garlic), (d) *Acacia arabica* (babul), and (e) *Aegle marmelos* (bel).

**Figure 2:** Acarbose % inhibition.

**Figure 3:** PHF showing maximum effects (hot water extract).

**Figure 4:** PHF showing moderate inhibitory effect (ethanol extract).

**Figure 5:** PHF showing moderate inhibitory effect (cold water extract).

**Figure 6:** PHF showing moderate inhibitory effect (benzene extract).

**Figure 7:** PHF showing moderate inhibitory effect (hexane extract).

**Figure 8:** (a) PHF showing the DPPH radical scavenging activity. (b) PHF showing H_2_O_2_ decomposition activity (GTA method). (c) PHF showing dose dependent antioxidant activity (TBARS method).

**Table 1:** The herbal plant composition is listed.

Plant name	Synonyms	Family	Parts of a plant used	Mass (g)
*Azadirachta indica*	Neem	Maliaceae	Leaves	25
*Aloe barbadensis*	Aloe vera	Liliaceae	Gel	25
*Allium sativum*	Garlic	Amaryllidaceae	Rhizome	25
*Acacia arabica*	Babul	Fabaceace	Seeds	25
*Aegle marmelos*	Bel or bilva	Rutaceae	Leaves	25

**Table 2:** Qualitative phytochemical screening.

Test	Hexane extract	Chloroform extract	Benzene	Ethanol extract	Cold water extract	Hot water extract
Carbohydrate	+	+	+	+	+	+
Glycosides	+	+	+	−	+	+
Alkaloids	−	−	−	−	−	+
Steroids	+	+	+	−	+	−
Terpenoids	−	−	−	+	−	+
Flavonoids	−	−	−	−	−	−
Phenol	+	+	+	+	+	+
Tannins	−	−	−	+ (G)	−	+ (G)
Saponins	−	−	−	+	−	−

where + sign indicates present, − sign indicates absent, and G indicates green colour.

**Table 3:** IC50 value of acarbose on alpha-amylase inhibition.

Standard drug	Concentration	% inhibition	IC50 value
Acarbose	10	15.65	90.35 ± 0.20
	20	19.42	
	40	26.33	
	60	35.27	
	80	45.60	
	100	55.30	

**Table 4:** PHF showing maximum effects (hot water extract).

Polyherbal formulation	Extract	Concentration	% inhibition	IC50 value
PHF	Hot water extract	10	20.4	48.98 ± 0.31
		20	38.2	
		40	47.1	
		60	56.7	
		80	67.7	
		100	79.5	

**Table 5:** PHF showing moderate inhibitory effect (ethanol extract).

Polyherbal formulation (PHF)	Extract	Concentration	% inhibition	IC50
PHF	Ethanol extract	10	14.6	69.42 ± 0.25
		20	23.5	
		60	30.2	
		80	39.6	
		100	68.6	

**Table 6:** PHF showing moderate inhibitory effect (cold water extract).

Polyherbal formulation (PHF)	Extract	Concentration	% inhibition	IC50 value
**PHF**	Cold water	**10**	**23.3**	90.55 ± 0.35
		**20**	**32.1**	
		**40**	**35.2**	
		**60**	**38.4**	
		**80**	**47.1**	
		**100**	**53.4**	

**Table 7:** PHF showing moderate inhibitory effect (benzene extract).

Polyherbal formulation (PHF)	Extract	Concentration	% inhibition	IC50 value
PHF	Benzene	**10**	**38.17**	**72.86** ± **0.28**
		**20**	**39.9**	
		**40**	**44.7**	
		**60**	**47.4**	
		**80**	**50.1**	
		**100**	**55.9**	

**Table 8:** PHF showing moderate inhibitory effect (hexane Extract).

Polyherbal formulation (PHF)	Extract	Concentration	% inhibition	IC50 value
PHF	Hexane	**10**	**9.6**	**142** ± **1.8**
		**20**	**16.3**	
		**40**	**25.6**	
		**60**	**29.4**	
		**80**	**31.2**	
		**100**	**36.6**	

**Table 9:** PHF showing the DPPH radical scavenging activity.

Concentration	% inhibition ± SD	
	Ascorbic acid	PHF
50 *μ*g/ml	50 ± 0.01^a^	46.1 ± 0.025^b^
100 *μ*g/ml	61.5 ± 0.05^b^	57.1 ± 0.02^a^
150 *μ*g/ml	70.1 ± 0.1^a^	63.2 ± 0.01^b^
200 *μ*g/ml	78.2 ± 0.02^b^	72.3 ± 0.02^a^
250 *μ*g/ml	81.2 ± 0.5^b^	77.2 ± 0.05^b^

Each value represents the mean ± SD, statistical significance compared with control (a: *p* < 0.01; b: *p* < 0.001).

**Table 10:** PHF showing H_2_O_2_ decomposition activity (GTA method).

Concentration	% inhibition ± SD	
	Ascorbic acid	PHF
50 *μ*g/ml	**30.1** ± **0.02**^**a**^	**23.2** ± **0.02**^**a**^
100 *μ*g/ml	**50.2** ± **0.05**^**b**^	**38.1** ± **0.023**^**a**^
150 *μ*g/ml	**55.3** ± **0.05**^**b**^	**42.3** ± **0.04**^**b**^
200 *μ*g/ml	**60.2** ± **0.03**^**a**^	**51.1** ± **0.03**^**b**^
250 *μ*g/ml	**80.2** ± **0.025**^**b**^	**78.2** ± **0.05**^**b**^

Each value represents the mean ± SD, statistical significance compared with control (a: *p* < 0.01; b: *p* < 0.001).

**Table 11:** PHF showing dose-dependent antioxidant activity (TBARS method).

Concentration	% inhibition ± SD	
	Ascorbic acid	PHF
50 *μ*g/ml	17.2 ± 0.02^a^	28.3 ± 0.02^b^
100 *μ*g/ml	45.2 ± 0.03^b^	39.2 ± 0.03^a^
150 *μ*g/ml	59.3 ± 0.04^a^	46.2 ± 0.04^b^
200 *μ*g/ml	78.2 ± 0.03^b^	61.1 ± 0.02^a^
250 *μ*g/ml	85.1 ± 0.04 ^b^	76.2 ± 0.03^b^

Each value represents the mean ± SD, statistical significance compared with control (a: *p* < 0.01; b: *p* < 0.001).

## Data Availability

All data used to support the findings of this study are included within the article.
